# Big Data Fusion Method Based on Internet of Things Collection

**DOI:** 10.1155/2022/1835309

**Published:** 2022-04-25

**Authors:** Tianrong Zhang, Hongying Li, Tian Jin, Fengjun Hu

**Affiliations:** ^1^Zhejiang Shuren University, Hangzhou, Zhejiang 310000, China; ^2^Zhejiang A&F University, Hangzhou, Zhejiang 311300, China

## Abstract

With the development of information collection technology, the data that people need to deal with are also increasing, which brings problems such as isomerization of data types, poor data quality, and fast data generation speed. At present, as an important method of data fusion technology, data fusion method based on deep learning has become an effective way of data fusion under the background of big data, which has important research significance. There is a problem with heterogeneous data types between time series data and text data, and it is difficult to fuse them effectively by traditional data fusion methods. In order to make full use of the information contained in text data and improve the accuracy of time series prediction, this paper proposes a data fusion model based on FC-SAE. In this model, GloVe and CNN are used to extract the features of text data, FC neural network is used to extract the potential features of time series data, and then, the SEA model is used to fuse the data, which fully discovers the relationship between data and greatly improves the prediction accuracy.

## 1. Introduction

Now, the ecological environment has been seriously affected, and the integration of ecological data is conducive to solving ecological and environmental problems. In this paper, a rotating forest algorithm is proposed to solve the problem of data fusion [1]. The model proposed in this paper solves the problem of data fusion well. Using the nonlinear mapping ability of neural network, the parallel processing of large-scale data is realized, and the fusion of multisource heterogeneous data is completed [2]. The effectiveness and usability of the convergence phase are of great significance for developers to improve the convergence [3]. This paper proposes a deep learning data fusion model to solve the traffic jam problem. The applicability of the model in traffic problems is obtained [4]. This paper proposes a data fusion method to improve the level of intelligent retrieval. The research shows that this method has obvious advantages in information recall and recall rate [5]. This paper studies how big data fusion mode method can effectively use big data to evaluate the relationship between them, and the effective evaluation rate is as high as 80% [6]. Deep learning is an advanced abstraction of modeling data, which is a branch of machine learning [7]. Deep learning uses a backpropagation algorithm to command machines to change their internal entries, thus discovering complex structures in large data sets [8]. This paper shows how to solve the research problems by training the deep network of learning features and how to share the representation learning patterns and evaluate them on a specific task [9]. In this paper, through a series of experimental studies, it is proved that deep learning can solve the problem of face recognition well. Face recognition tasks increase the differences between people by extracting verification features from different identities, while face verification tasks reduce the differences between people by combining verification features extracted from the same identity, which are necessary for face recognition [10]. Through a large number of systematic experiments, this paper shows why traditional methods cannot explain the generalization ability of large neural networks [11]. This paper briefly describes the application research of deep learning in each field. The most advanced technology at present is summarized, and the future research direction is given [12]. Although deep learning is widely used, it cannot capture the uncertainty of the model. Although the Bayesian model can reason the uncertainty of the model, its computational cost is very high [13]. The specificity of DNA binding to protein can be determined by deep learning technology. Experiments show that this algorithm is more excellent than other algorithms [14]. In this paper, an algorithm is created by deep learning, which can be applied to the field of medical imaging [15]. When the deep learning model uses data collection, it can obtain the complex underlying structure of the data system, especially for large data sets and high-dimensional data sets. When the features are complex, the data set collects more information and can retain more feature values.

## 2. Main Methods of Data Fusion

### 2.1. Weighted Average Method

This method directly processes the original information collected by the sensing nodes. Its fusion idea is to get the weight coefficient of each sensing node according to certain algorithm rules and then weigh the redundant data of each sensing node according to the weight, and the result is to calculate the weighted average value of the data collected by sensing nodes, which makes the data more accurate and concise. The advantages of this fusion method are easy and intuitive, but the main disadvantages are as follows: there is no deletion of redundant information, which will lead to an increase in computing energy consumption.

### 2.2. Bayesian Reasoning

Bayesian estimation is a common uncertainty reasoning method, and it is also a statistical fusion method. It usually uses the detection area and prior knowledge to determine the target in the detection area. It can fuse nodes and information, and then get the hypothetical posterior probability.

### 2.3. Kalman Filtering Method

Most of these fusion methods appear in dynamic topology, which can fuse perceptual data and remove redundant data in real time. This method uses the linear combination to get the final fusion result, which is an estimate with low accuracy. When necessary, it also needs to introduce the concept of adaptive.

### 2.4. Neural Network Method

Neural network structure is a network model of general fusion methods, and fuzzy reasoning is generally adopted as the main idea of data fusion. It firstly establishes a fuzzy reasoning mechanism based on the sample data of the sensing nodes and then fuses the data, so it has good fault tolerance and robustness.

### 2.5. Fuzzy Logic Reasoning

This method can deal with uncertain information reasonably. In addition, the information processing method of this method is close to human thinking, so it often appears in higher-level fusion operations. It also has many disadvantages, such as subjective description of data.

  Weighted average method: easy to understand, good real time, suitable for changeable scenes.
  Kalman filtering method: It is suitable for linear system, so that the system does not need a lot of data storage and calculation, and can be processed in real time.
  Bayesian inference method: concise, medium computation, and good effect of related events.
  Template method: good effect in non-real-time environment.
  Fuzzy theory: It can solve the problem of information or decision conflict and realize the information fusion between subjective and objective.

## 3. Fusion Model Framework Based on FC-SAE

FC-SAE model mainly includes text feature extraction, time series modeling, and heterogeneous data feature fusion. Text feature extraction module mainly preprocesses text data, mines semantic relations through the GloVe word embedding algorithm, and extracts features at different abstract levels by convolution neural network; neural network is used to model time series. Heterogeneous data feature fusion module uses the encoder of sparse automatic encoder to fuse text features and time series features and extract the fused features.

### 3.1. Text Feature Extraction

When the text data are converted into text sequence, it enters the word embedding layer. The essence of word embedding is to make words and vectors correspond one by one. To get the relationship in embedding space, we only need to calculate the distance between vectors. In FC-SAE model, GloVe word embedding model is used for word embedding operation.

The basic idea of this model is to decompose the global vocabulary matrix and train the word vectorization model with window. The training process of GloVe word embedding model mainly includes constructing word co-occurrence matrix and training word vector.

GloVe model constructs a word co-occurrence matrix *X*. Suppose the corpus is “sheisthemostlovelyperson,” and there are six words in the corpus: she, is, the, most, lovely, person. The window information is shown in Table 1.

Take window 3 as an example, there are the following formulas:

(1) $$\begin{array}{c} X_{\text{the,is}}=X_{\text{the,is}}+1, \end{array}$$

(2) $$\begin{array}{c} X_{\text{the,most}}=X_{\text{the,most}}+1. \end{array}$$

The co-occurrence matrix *X* can be obtained according to the above method. According to the co-occurrence matrix, the probability of occurrence of the word *J* in the context of the word *I* can be obtained, and the calculation is as shown in formula (3)

(3) $$\begin{array}{c} P_{ij}=P\left(j|i\right)=\frac{X_{ij}}{X_{i}}. \end{array}$$

In the formula, *X*_*i*_=∑_*k*_*X*_*ik*_. The relation of the words *I*, *J*, and *K* can be expressed as

(4) $$\begin{array}{c} {\text{radio}}_{i,j,k}=\frac{P_{ik}}{P_{jk}}. \end{array}$$

When the value of radio_*i*,*j*,*k*_ is small, the correlation between *J* and *K* is high, while the correlation between *I* and *K* is low. When the value of radio_*i*,*j*,*k*_ tends to 1, while the word *I* is related to the word *K* and the word *J* is also related to the word *K*, or while the word *I* is not related to the word *K* and the word *J* is not related to the word *K*. Therefore, radio_*i*,*j*,*k*_ can better measure the correlation between words.

The purpose of GloVe model is to construct a function $F\left(v_{i},v_{j},{\tilde{v}}_{k}\right)$ by using word vectors *v*_*i*_, *v*_*j*_, and ${\tilde{v}}_{k}$, so that the value of this function is as close as possible to (*P*_*ik*_/*P*_*jk*_). The model loss function is shown in formula (5)

(5) $$\begin{array}{c} J=\sum_{i,j}^{N}f\left(X_{i,j}\right){\left(v_{i}^{T}{\tilde{v}}_{j}+b_{i}+b_{j}-\log\left(X_{ij}\right)\right)}^{2}, \end{array}$$

where *N* is the number of words, and the co-occurrence matrix *X* is the *N* × *N* matrix; *X*_*ij*_ denotes the number of times the word *I* and the word *J* appear in the same window; *v*_*i*_^*T*^ denotes the transposition of the word vector corresponding to the word *I*; ${\tilde{v}}_{j}$ denotes the word vector corresponding to the word *J* when the word *J* is the central word of the context; *b*_*i*_ and *b*_*j*_ are bias terms; and *F* is a custom weight function. The common form of weight function is given by

(6) $$\begin{array}{c} f\left(x\right)=\left\{\begin{array}{cc} {\left(\frac{x}{x_{\max}}\right)}^{\alpha }, & x<x_{\max},\\ 1, & x\geq x_{\max}, \end{array}\right) \end{array}$$

where *x*_max_=100, *α*=0.75, and word vector and word vector model can be obtained by minimizing loss function.

We use convolution neural network to further extract the features of text data. The word vector matrix *X*[*i* : *j*] obtains a feature map *C* by convolution operation through a convolution layer and obtains a maximum value $\hat{C}$ in the feature map through a maximum pooling layer, which represents the most important feature. The output feature *Z*_text_ of the word vector matrix is obtained under the action of a plurality of convolution kernels, and the process is shown in formulas (7)–(10):

(7) $$\begin{array}{c} C_{i}=f\left(wX\left[i:j\right]+b\right), \end{array}$$

(8) $$\begin{array}{c} C=\left[C_{1},C_{2},\ldots ,C_{n}\right], \end{array}$$

(9) $$\begin{array}{c} \hat{C}=\max\left\{C\right\}, \end{array}$$

(10) $$\begin{array}{c} Z_{\text{text}}=\left[{\hat{C}}_{1},{\hat{C}}_{2},\ldots ,{\hat{C}}_{m}\right], \end{array}$$

where *n* is the number of feature mappings and *m* is the number of convolution kernels. This model can obtain the variable length mode of input text with arbitrary length.

### 3.2. Time Series Modeling Based on Full Connection Layer

Deep learning methods commonly used in time series prediction include RNN, LSTM network, and fully connected network. LSTM is the most commonly used deep learning algorithm for time series prediction because it can well obtain the medium- and long-term dependence of time series data. Detrending data can largely eliminate the need for long-term dependencies, which makes LSTM inferior to FC. Therefore, this paper uses FC to model time series.

The calculation steps of the fully connected network output are as follows:

First calculate the weighted sum, as shown in the following formula:

(11) $$\begin{array}{c} s_{b}=\sum_{b=1}^{n}\left(W_{ab}X_{a}+\theta_{b}\right). \end{array}$$

In the above formula, *W*_*ab*_ represents the connection weight of nodes *a* to *b*, *θ*_*b*_ is the offset term of the *b* hidden node, and *X*_*a*_ is input. The output of each node is calculated according to formulas (12)–(14):

(12) $$\begin{array}{c} S_{b}=\text{sigmoid}\left(s_{b}\right)=\frac{1}{\left(1+\exp\left(-s_{b}\right)\right)},\;b=1,2,\ldots ,h, \end{array}$$

(13) $$\begin{array}{c} o_{k}=\sum_{b=1}^{h}\left(W_{bk}S_{b}+\theta_{k}\right),\;k=1,2,\ldots ,m, \end{array}$$

(14) $$\begin{array}{c} O_{k}=\text{sigmoid}\left(o_{k}\right)=\frac{1}{\left(1+\exp\left(-o_{k}\right)\right)},\;k=1,2,\ldots ,h, \end{array}$$

where *W*_*bk*_ is the connection weight between the *b*-th and *k*-th output nodes, and *θ*_*k*_ is the offset term of the *k*-th output node.

In FC-SAE data fusion model, the form of delayed observation is used as the fixed input vector, as shown in following formula:

(15) $$\begin{array}{c} Z_{ts}=f\left(wT+b\right), \end{array}$$

where *Z*_*ts*_ is the time series feature, and *T*=(*t*_1_, *t*_2_,…*t*_*L*_) and *L* are the lag observation lengths.

### 3.3. Feature Fusion of Heterogeneous Data

At present, in the research of data fusion based on deep learning, most researchers use feature mosaic and full connection layer to fuse the extracted features. Although this fusion method is very simple, it cannot fully mine the relationship between data. FC-SAE model takes the sparse automatic encoder as the fusion module, which can fully mine the relationship between time series data and text data while retaining the maximum amount of information, so as to obtain the shared feature representation of data.

The sparse automatic encoder is a deep learning model without supervision and management. In FC-SAE model, firstly, data features and sequence features are combined to obtain *x*, and then, the combined features *x* are input into SAE fusion model, output through hidden layer and nonlinear mapping, represented by *y*, and finally mapped back to *x*′. The above is the encoding and decoding process, which is represented by

(16) $$\begin{array}{c} y=h\left(Wx+b\right), \end{array}$$

(17) $$\begin{array}{c} x{}^{\prime }=h{}^{\prime }\left(W{}^{\prime }y+b{}^{\prime }\right). \end{array}$$

In the above formula, *H* represents the activation function of the encoder, *H* represents the activation function of the decoder, *W* represents the weight matrix of the encoder, *W* represents the weight matrix of the decoder, *B* represents the bias term of the encoder, and *B* represents the bias term of the decoder. The loss function can be expressed by formulas (18)–(20):

(18) $$\begin{array}{c} \text{Cost}=\frac{1}{n}\sum_{k}{\left(x_{k}-x_{k}^{\prime }\right)}^{2}+\frac{\lambda }{2}{\sum_{l}^{L}\sum_{j}^{n}\sum_{i}^{k}\left({\left(w\right)}_{ij}^{l}\right)}^{2}+\beta \psi_{\text{sparsity}}, \end{array}$$

(19) $$\begin{array}{c} \psi_{\text{sparsity}}=\sum_{i}\rho \;\log\frac{\rho }{{\hat{\rho }}_{i}}+\left(1-\rho \right)\log\frac{1-\rho }{1-\rho_{i}}, \end{array}$$

(20) $$\begin{array}{c} {\hat{\rho }}_{i}=\frac{1}{n}\sum_{j=1}^{n}y_{i}\left(x_{j}\right), \end{array}$$

where *L* is the number of hidden layer nodes, *n* is the number of data samples, and *k* is the input vector dimension. *λ* and *β* are given coefficients, which control the weighted coefficient regular term and the sparse regular term, respectively. ${\hat{\rho }}_{i}$ is the average activation value of neurons in hidden layer, and *ρ* is the sparsity parameter.

## 4. Experimental Results and Analysis

### 4.1. Data Sets and Data Preprocessing

The selection of time series data in this experiment is consistent with that in the previous chapter. Meteorological data are a public data set of the National Oceanic and Atmospheric Administration of the United States, which has 13 characteristics. The event text data are obtained from Barclays Center official website. The data set contains 751 event description text data, each of which includes title, time, and event description. The event presence data are generated from the event text data, and the value is 1 on the date when an event occurs and 0 on the date when no event occurs. Some data of the above experimental data set are shown in Tables 2–4.

When dealing with taxi data, the original data are added first to get daily travel data. In order to reduce the impact on the data in the later period, the data are processed by trend, which makes the model pay more attention to the fluctuation of the data itself and improves the prediction effect. The preprocessing operation of meteorological data is to normalize the data. The preprocessing of text data is conventional text preprocessing, including HTML tag deletion, lowercase conversion, root, deletion of stop words, and prepositions.

### 4.2. Experimental Design

FC-SAE model uses GloVe word embedding model and CNN neural network to extract features from text data in which CNN includes three convolution layers and three pooling layers, and ReLU function is used as activation function; a two-layer FC neural network with 100 neurons and 50 neurons is used to model the time series. Tanh function is used as activation function, and the input data are standardized before FC layer input. SAE is used as the fusion model, and Adam is used to optimize the model parameters.

This paper compares the nonlinear time series forecasting model with FC-SAE model and concludes that FC-SAE model has more advantages in forecasting. In addition, FC-SAE model is replaced by LSTM-SAE model, and its effectiveness is verified. Then, the contribution of information from different sources to data fusion is evaluated. This paper also analyzes the incremental experiments of FC-SAE model and LSTM-SAE model. Finally, in order to compare the impact of different fusion strategies on the prediction results, under the condition of complete model, the fusion model based on full connection layer is compared with the fusion model based on the sparse automatic encoder.

### 4.3. Analysis of Experimental Results

In this paper, root mean squared error (RMSE), mean absolute error (MAE), and goodness-of-fit R2 are selected to evaluate the proposed model, as shown in formulas (21)–(23):

(21) $$\begin{array}{c} \text{MAE}=\frac{1}{N}\sum_{n=1}^{N}\left|y_{n}-{\hat{y}}_{n}\right|, \end{array}$$

(22) $$\begin{array}{c} \text{RMSE}=\sqrt{\frac{1}{N}\sum_{n=1}^{N}{\left(y_{n}-{\hat{y}}_{n}\right)}^{2}}, \end{array}$$

(23) $$\begin{array}{c} R^{2}=1-\frac{\sum_{n-1}^{N}{\left(y_{n}-{\hat{y}}_{n}\right)}^{2}}{\sum_{n-1}^{N}{\left(y_{n}-\bar{y}\right)}^{2}}, \end{array}$$

where *N* represents the amount of data in the test set, *y*_*n*_ represents the true value of the nth instance, and ${\hat{y}}_{n}$ represents the predicted value of the nth instance. Both MAE and RMSE can reflect the deviation degree of the two values. The smaller the two values, the better the prediction effect, and RMSE is the most sensitive to outlier data. The fitting degree of the model can be measured by *R*, and the larger the value, the better the fitting effect of the model.

#### 4.3.1. Comparison with Other Time Series Forecasting Methods

Firstly, this paper compares the differences in MAE, RMSE, and R2 indexes among FC-SAE model and SVR model, GP model, LSTM neural network, and LSTM-SAE model, as shown in Table 3. The results show that LSTM is not the best choice for the time series prediction in this paper. And by adjusting the parameters of LSTM-SAE model, it cannot achieve the performance of FC-SAE model. The results also verify the conclusions of early studies on LSTM. Compared with SVR algorithm, GP algorithm, and LSTM algorithm, FC-SAE model has improved by 1.3%, 5.3%, and 6.6% in MAE index; 1.8%, 5.4%, and 4% in RMSE index; and 1.8%, 6.6%, and 7.7% in R2 index, respectively, which has obvious advantages. From the experimental results in Table 3, it can be seen that FC-SAE model and SVR model are better methods in this research field, and the time series prediction method based on data fusion has obvious advantages over the traditional time series prediction method, as shown in Figure 1 and Table 5.

#### 4.3.2. Comparative Experiment of Multisource Heterogeneous Data Fusion

In order to further analyze the influence of each data on the fusion effect, the incremental analysis method is selected for the experiment. Firstly, only time series is modeled, and then, meteorological data, event existence data, and event text description data are added in turn. The results are shown in Figures 2–4.

Looking at Figures 2–4, we can see that the best way to improve the prediction results of time series is to introduce meteorological data. From an empirical point of view, bad weather conditions will change people's travel mode, which is consistent with our experimental results. The event presence data (*E*) have the greatest influence on the prediction results. After introducing the event presence data, the MAE index and RMSE index of FC-SAE algorithm are reduced by 17.1% and 12.6%, respectively. The MEA algorithm decreased by 17%, and the RMSE algorithm decreased by 15.3%. Although the introduction of event existence data has significantly improved the prediction effect of FC-SAE algorithm and LSTM-SAE algorithm, it is impossible to judge the real impact of events on prediction results without further analysis of the information contained in event description. In this paper, the text description of events is introduced into time series prediction through GloVe word embedding model and convolution neural network. Experimental results show that the MAE index of FC-SAE algorithm decreases from 99.3 to 95.9, RMSE index also decreases from 140.3 to 135.8, and R2 increases from 0.599 to 0.626 after combining event text description data (TS) with other data. In the same way, the MAE and RMSE of LSTM-SAE algorithm are reduced by 6.6% and 2.2%, respectively. Therefore, the introduction of different data has different effects on the prediction results. The event existence data have a greater impact, and the event description text data have a certain degree of improvement on the prediction results, but it is not as obvious as the former.

#### 4.3.3. Comparative Experiment of Fusion Methods

In order to verify the effectiveness of SAE fusion model, this paper compares FC-SAE model and LSTM-SAE model with the models using full connection layer fusion: FC-FC model and LSTM-FC model, and the results are shown in Table 4. Through observation, we can conclude that SAE model is obviously higher than FC model in data fusion prediction. Compared with FC-FC model, the MAE index and RMSE index of FC-SAE model decreased by 1.7% and 2.3%, respectively, while the MAE index and RMSE index of LSTM-SAE model decreased by 2.1% and 2.2%, respectively, compared with LSTM-FC algorithm. During the experiment, it is found that the advantage of using SAE model for fusion is that it can fully mine the correlation between time series data and text data, while retaining the maximum amount of information. The experimental results verify that SAE fusion model performs better in heterogeneous data fusion than full connection layer, as shown in Figure 5 and Table 6.

This chapter takes common time series data and text data as data sources, establishes multisource heterogeneous data fusion model based on FC-SAE, studies the fusion of time series data and text data, and discusses the influence of event text data on time series prediction. By comparing FC-SAE data fusion model with other popular time series prediction methods, it is proved that FC-SAE data fusion model has better prediction accuracy; the comparative experiment of multisource heterogeneous data fusion proves that the error of time series prediction results can be effectively reduced by multisource heterogeneous data fusion, and different data have different influences on prediction results. In addition, the comparison experiments of fusion methods show the influence of different fusion strategies on the prediction results, and the results show that SAE fusion model has better fusion performance than FC fusion model.

## 5. Conclusion

This paper presents a multisource heterogeneous data fusion model based on FC-SAE. This paper presents a data fusion model based on FC-SAE to solve the data fusion processing of time series data and text data. In this model, FC neural network is used to extract the features of time series, GloVe and CNN are used to extract the features of text data, and finally, SAE model is used to fuse the features of data. This model solves the problem that data fusion is difficult caused by data type differences. By analyzing the experimental results, we find that FC-SAE model can make the time series achieve the best accuracy in heterogeneous data fusion. Moreover, through the analysis of incremental experiments, we can know the influence of different data on the fusion results in data fusion. Finally, by comparing different fusion strategies, it is proved that the fusion effect of SAE model is better than that of full connection layer fusion.

## Figures and Tables

**Figure 1:** Comparison diagram of various models.

**Figure 2:** MAE evaluation index of multisource heterogeneous data fusion experiment.

**Figure 3:** RMSE evaluation index.

**Figure 4:** *R* evaluation index of multisource heterogeneous data fusion experiment.

**Figure 5:** Comparison diagram of fusion methods.

**Table 1:** Window information.

Numbering	Head word	Content
1	she	she is
2	is	she is the
3	the	is the most
4	most	the most lovely
5	lovely	most lovely
6	person	lovely person

**Table 2:** Taxi travel data.

Date	Hour	Minute	Pickups
2009/1/1	0	0	2
2009/1/1	0	1	15
2009/1/1	1	0	13
2009/1/1	2	0	19

**Table 3:** Meteorological data.

Date	min_te	max_te	wi_sp	wi_g	vis	pers	pptn	snow_d	fog	rain	s_ice	ts
2009/1/1	15.1	26.1	11.6	32.1	10	1015.5	0.04	999.9	0	0	0	0
2009/1/2	21.9	33.1	5.6	19	9.3	1011	0	999.9	0	0	1	0
2009/1/3	30	37.9	7.7	20	10	1007.6	0	999.9	0	0	0	0
2009/1/4	25	42.1	7.3	17.1	10	1013.1	0	999.9	0	0	0	0
2009/1/5	37.9	43	6.3	14	10	1009.3	0	999.9	0	0	0	0

**Table 4:** Event text description data.

Date	start_time	Title	URL	Description
2013/2/22	2013-02-33 19:30:00	Brooklyn Nets vs Houston Rockets	https://www.barclayscenter.com/events/deta%20il/brooklyn-nets-vshouston-rockets	Jeremy James hardenly makes their only appearance when Houston rocket travel what should high octane arrival revamped rocket have been racing all season net more provides style
2015/10/9	2015/10/9 19:30	New York Islanders vs. Chicago Blackhawks	https://www.barclayscenter.com/events/deta%20il/new-york-islandersvs-chicagoblackhawks	make dinner reservation today by calling and emailing (email protected) click here to see event menu club restaurant American express
2015/3/20	2015/3/20 19:30	Brooklyn Nets vs. Milwaukee Bucks	https://www.barclayscenter.com/events/deta%20il/brooklyn-nets-vsmilwaukee-bucks-3-20-15	Nan

**Table 5:** Model comparison.

Method	MAE	RMSE	*R* ^2^(×100)
SVR	97.2	138.3	61.5
GP	101.2	143.6	58.7
LSTM	102.7	141.5	58.1
LSTM-SAE	98.3	139.7	61.1
FC-SAE	95.9	135.8	62.6

**Table 6:** Comparative experiment of fusion methods.

Method	MAE	RMSE	*R* ^2^(×100)
FC-SAE	95.9	135.8	62.6
FC-FC	97.6	139.1	62.2
LSTM-SAE	98.3	139.7	61.1
LSTM-FC	100.4	142.9	59.5

## Data Availability

The experimental data used to support the findings of this study are available from the corresponding author upon request.
